The article "Better short-term efficacy of treating severe flail chest with internal fixation surgery compared with conservative treatments" was published in 2015. Journal: Eur J Med Res.

# Better short-term efficacy of treating severe flail chest with internal fixation surgery compared with conservative treatments

**DOI:** 10.1186/s40001-015-0146-0

**Published:** 2015-05-24

**Authors:** Jing-Qing Xu, Pei-Li Qiu, Rong-Guo Yu, Shu-Rong Gong, Yong Ye, Xiu-Ling Shang

**Affiliations:** SICU, Fujian Provincial Hospital, Fujian Medical University Affiliated Provincial Teaching Hospital, Fuzhou, 350001 China

**Keywords:** Flail chest, Surgery, Internal fixation, Trauma, Conservative treatment

## Abstract

**Background:**

The objective of the study is to provide evidence for selecting the best treatment approach for severe flail chest by comparing surgical and conservative treatments.

**Methods:**

This is a retrospective study in which 32 patients with severe flail chest were treated in the Fujian Provincial Hospital (China) between July 2007 and July 2012 with surgical internal rib fixation (*n* = 17) or conservative treatments (*n* = 15). Mechanical ventilation time, intensive care unit (ICU) stay time, pulmonary infection, antibiotic treatment duration, acute physiology and chronic health evaluation II (APACHE II) scores 7 and 14 days after trauma, rate of tracheostomy, and rate of endotracheal re-intubation were compared.

**Results:**

One patient died in the conservative treatment group. Better short-term outcomes were observed in the surgery group, such as total mechanical ventilation time (10.5 ± 3.7 vs. 13.7 ± 4.4 days, *P* = 0.03), ICU stay (15.9 ± 5.0 vs. 19.6 ± 5.0 days, *P* = 0.05), pulmonary infection rate (58.8 % vs. 93.3 %, *P* = 0.02), and APACHE II scores on the 14th day (6.5 ± 3.8 vs. 10.1 ± 4.7, *P* = 0.02). No difference was observed in the therapeutic time of antibiotics, rate of tracheostomy, and the rate of endotracheal re-intubation between the two groups.

**Conclusions:**

Results suggest that internal fixation surgery resulted in better outcomes in the management of severe flail chest compared with conservative treatments.

## Background

Blunt thoracic trauma is one of the most common traumas and results in flail chest in about 10 % of cases [1]. Flail chest occurs when three or more adjacent ribs are fractured in at least two places, creating a chest wall segment that moves paradoxically from the remaining chest wall. Flail chest is associated with significant morbidity and mortality (10–15 % mortality) [1]. Loss of chest wall integrity could induce lobar atelectasis and alveolar collapse; pain and accumulation of secretions could further aggravate pulmonary atelectasis, decrease tidal volume, and induce hypoventilation. The pathophysiology of severe flail chest is rooted in the combination of an underlying pulmonary parenchymal contusion and the paradoxical motion of the flail segment that results in an inability to generate negative intrathoracic pressure leading to hypoventilation of the damaged area. Compensatory mechanisms in response to hypoventilation include pulmonary vasoconstriction which leads to shunting, leading to pulmonary hypertension. For patients with pulmonary parenchyma injuries, hemothorax and/or pneumothorax could also impair generate negative intrathoracic pressure and contributes to the ventilation/perfusion mismatch [2]. Therefore, flail chest may induce respiratory distress, hyoxemia, and/or hypercapnia, and the patient may need mechanical ventilation. The mortality rate also increases substantially with age and the number of fractured ribs [3].

Two treatment approaches are available for flail chest: surgical and conservative [4, 5]. Standard conservative treatment mainly requires positive pressure ventilation, along with analgesia, bronchoalveolar lavage via fiberoptic bronchoscopy, local pressure bandaging of the loose thoracic wall, and suspension traction of the ribs [6]. Conservative treatment could result in deformities of the thoracic wall, which could result in chronic pulmonary insufficiency and pleuritic chest pain [7]. And the bandages limited paradoxical chest wall segment also made the patients to remain supine for a long period of time, which led to underlying complications. However, despite favorable outcomes, surgery is associated with some criticisms, such as unknown long-term outcomes, surgical trauma, wound infections, and technical anatomical difficulties [5, 8, 9]. Besides that, great advances in mechanical ventilation during recent years also help the patients of conservative treatment out of threats from respiratory failure earlier. A recent meta-analysis supports the use of surgery for flail chest but underlines the need for an adequately powered clinical trial [10]. And a recent prospective randomized study of 46 patients reported favorable outcomes when using surgery to treat flail chest [11]. Nevertheless, the correct treatment approach is still controversial [5]. In addition, since there is a lack of knowledge about the operation indications and benefits from surgery and the new technologies, physicians’ surgery awareness is extremely low [12].

Therefore, there is still a controversy about whether flail chest should be treated with surgical or conservative treatment. In the present study, we retrospectively analyzed the data from 32 patients with severe flail chest that had been treated with the conservative or surgical approach in our hospital between July 2007 and July 2012. We aimed to provide evidence for choosing the best treatment method for patients with severe flail chest.

## Methods

### Subjects

Patients with multiple rib fractures who had been treated in our hospital between July 2007 and July 2012 were included. The patients were divided into two groups, namely the conservative and the surgery groups, according to the treatment they originally received. Patients in the conservative group received standard conservative treatment, while the patients in the surgical group underwent surgical internal fixation. The present study was approved by the ethics committee of the Fujian Provincial Hospital.

### Inclusion and exclusion criteria

Inclusion criteria were: 1) four or more rib fractures; 2) abnormalities of the thoracic cage and paradoxical breathing; and 3) requirement for mechanical ventilation during treatment. Exclusion criteria were: 1) age <14 or >75 years; 2) severe craniocerebral trauma (Glasgow Coma Scale [GCS] score <8); 3) no spontaneous breath after high-level spinal cord injury; or 4) history of chronic cardiopulmonary disease.

### Treatment procedures

Physical examinations, laboratory assays (including arterial blood gas analysis), and imaging (including spiral chest CT scanning for 28 patients and chest X-ray for four) were performed for all patients. Electrocardiogram, intravenous infusion, and ventilator-assisted respiration were also performed according to the progress of emergency rescue. In addition, antibiotics, closed thoracic drainage, blood product infusion, wound debridement, fiberoptic bronchoscope-assisted airway secretion clearance, analgesia, sedation, and treatment of complications were performed if necessary.

In addition to the treatments described above, for the patients in the conservative group, non-surgical treatments included pressure bandaging and external fixation with pectoral girdle. For the patients in the surgery group, conventional rib fracture plating was performed [8].

Arterial blood gas analysis was performed as respiratory and ventilator parameters were changed in both the groups. Once hemodynamics was stable and no hypoxemia (FiO_2_ ≤ 40 %) or hypercapnia was found, spontaneous breathing trials were also performed to help accelerate ventilator weaning.

Internal fixation of rib fractures was performed as follows [8]. An incision was made at the center of the collapsed area of the thoracic cage after general anesthesia. Separation of the subcutaneous tissues was performed, and the fractured ends were exposed along the distribution of the muscles (resection of the muscle fibers was minimized during the process). To avoid damage to the intercostal arteries and nerves, the periosteum should be separated carefully. The fractured ends were pulled together and fixed with low-profile titanium-locking plates, and then a surgical drain was subcutaneously implanted.

### Data collection

Mechanical ventilation time, intensive care unit (ICU) stay time, pulmonary infection, therapeutic time of antibiotics, acute physiology and chronic health evaluation II (APACHE II) score 7 and 14 days after trauma, rate of tracheostomy, and rate of endotracheal re-intubation were collected and analyzed.

Injury severity scores (ISS) were calculated as the sum of squares of the highest abbreviated injury scale (AIS) score of three different body regions. The severity was classified according to the guidelines by Baker et al.: ISS <16 was classified as minor injury, ISS 16–24 was classified as severe injury, and ISS >25 was classified as critical injury. As for patients with an AIS equal to 6 in one or more regions, the ISS score was automatically set as 75 [13]. The mortality rate of patients with an ISS >20 is substantially increased, while which with ISS >50 is extremely high.

APACHE II scores were determined as originally described [14].

### Statistical analysis

SPSS 16.0 (SPSS Inc., Chicago, IL, USA) was used for statistical analysis. Continuous data were described as means ± standard divisions (SD) and analyzed using the Student’s *t*-test. Categorical data were analyzed using the chi-square test. *P*-values <0.05 were considered statistically significant.

## Results

### Clinical characteristics

Data from 363 patients with multiple rib fractures who have been treated in our hospital between July 2007 and July 2012 were reviewed; 41 patients met the inclusion criteria, but according to our exclusion criteria, 32 patients were enrolled in this study finally. Fifteen patients (12 males and 3 females; mean age of 39.0 ± 11.6 years, ranging from 18 to 58 years) received conservative treatments, while 17 patients (12 males and 5 females; mean age of 36.4 ± 13.5 years, ranging from 15 to 61 years) underwent surgery. The mean number of rib fractures was 7.4 ± 1.6 in the conservative group and 6.8 ± 2.1 in the surgery group. Eleven patients in the conservative group and 13 patients in the surgery group suffered from pulmonary injuries, and the mean ISS scores were 24.0 ± 8.0 and 21.8 ± 7.8, respectively. The mean APACHE II scores were 15.3 ± 7.2 and 13.7 ± 5.5 in the conservative and surgery groups, respectively. There was no significant difference in age, gender, number of rib fractures, rate of pulmonary contusion, ISS scores, and APACHE II scores between the two groups (Table 1). Therefore, the two groups of patients were comparable.

**Table 1:** Baseline patients’ clinical characteristics

	All patients (*n* = 32)	Group A (*n* = 15)	Group B (*n* = 17)	*P*-value
Age (year, mean *±* SD)	37.6 ± 12.5	39.0 ± 11.6	36.4 ± 13.5	0.727
Gender (male/female)	24/8	12/3	12/5	0.593
Number of rib fractures (mean *±* SD)	7.1 ± 1.9	7.4 ± 1.6	6.8 ± 2.1	0.336
Pulmonary injury	24	11	13	0.838
ISS score (mean *±* SD)	22.6 ± 8.0	24.0 ± 8.0	21.8 ± 7.8	0.879
APACHE II score at admission (mean *±* SD)	14.4 ± 6.3	15.3 ± 7.2	13.7 ± 5.5	0.461

One patient in the conservative group died from critical acute respiratory distress syndrome (ARDS) induced by a severe pulmonary infection. In the surgery group, no broken or loose metal plates and wound infections were observed.

### Treatment efficacy

There was a difference in the mean mechanical ventilation time between the two groups (conservative: 13.7 ± 4.4 vs. surgery: 10.5 ± 3.7 days, *P* = 0.033). Further analysis showed that for patients with pulmonary injuries, significantly shorter mechanical ventilation time was needed for the ones treated with surgical treatment (*n* = 13) compared with the ones treated with conservative treatments (*n* = 11; 10.4 ± 3.8 vs. 14.4 ± 5.0 days, *P* = 0.038). Mean time of ICU stay was 19.6 ± 5.0 and 15.9 ± 5.0 days for the patients in the conservative and surgery groups, respectively (*P* = 0.047). There was no difference in the mean antibiotic treatment duration between the two groups. Pulmonary infection was found in 14 (93.3 %) and 10 (58.8 %) patients in the conservative and surgery groups, respectively (*P* = 0.024). There was a statistical trend in the surgery group having fewer tracheotomies (2) than in the conservative group (6) (*P* = 0.066). There was no statistically significant difference in the rates of endotracheal re-intubation (conservative: 3/15 vs. surgery: 1/17, *P* = 0.288).

On average, the APACHE II score decreased by about 1.9 on the seventh day after admission compared with the score at admission in the conservative group and decreased by about 2.3 in the surgery group. The score decreased by 4.2 and 7.2 on the 14th day after admission in the conservative and surgery groups, respectively, compared with the score at admission. The changes in APACHE II scores showed that the condition improvements were significantly better in surgery group as time went by (Table 2).

**Table 2:** Patients’ clinical data

	Group A	Group B	*P-*value
Ventilation time (mean ± SD)	13.7 ± 4.4	10.5 ± 3.7	0.033
ICU stay (mean *±* SD)	19.6 ± 5.0	15.9 ± 5.0	0.047
Therapeutic time of antibiotics (mean *±* SD)	17.9 ± 6.7	14.9 ± 5.9	0.187
Pulmonary infection	14/15	10/17	0.024
Tracheostomy	6/15	2/17	0.066
Endotracheal re-intubation	3/15	1/17	0.288
APACHE II on the seventh day (mean *±* SD)	13.4 ± 5.8	11.4 ± 5.0	0.350
APACHE II on the 14th day (mean *±* SD)	10.1 ± 4.7	6.5 ± 3.8	0.021

For the patients in the surgery group, the surgeries were performed 3–15 days after admission (mean time: 6.5 days). To explore the effects of operation timing on the outcomes, the patients were classified into two subgroups, the early surgery group (time from trauma to operation was ≤5 days; 5 males and 2 females) and the late surgery group (time from trauma to operation was >5 days; 7 males and 3 females). Analysis showed that an early operation could further shorten the ventilation time compared with a late operation (7.9 ± 1.5 vs. 12.3 ± 1.7 days, *P* = 0.008).

## Discussion

The use of surgery for the treatment of flail chest is still controversial [5]. The aim of this study was to compare surgical vs. nonsurgical treatment for severe flail chest. Results showed that clinical outcomes were better in the surgery group, such as total mechanical ventilation time, ICU stay, pulmonary infection rate, and APACHE II scores on the 14th day. These results suggest that surgical treatment of severe flail chest resulted in improved short-term outcomes compared with a conservative treatment approach.

A prospective randomized clinical trial by Tanaka et al. [15] reported that the mean ventilation time in the surgical treatment group (10.8 ± 3.4 days) was significantly shorter than in the conservative treatment group (18.3 ± 7.4 days), and that ventilator weaning could be successfully performed 2.5 ± 3.2 days after operation for patients in the surgical treatment group. In the present study, the ventilation time was 13.7 ± 4.4 days in the conservative group, while the ventilation time was significantly shorter in the surgical group (10.5 ± 3.7 days). These results are consistent with those published in a recent meta-analysis [10]. Early ventilator weaning may reduce the stress caused by invasive endotracheal intubation and decrease the use of sedative-analgesic drugs but also significantly reduce the incidence of ventilator-associated pneumonia and in turn reduce the ICU stay and overall hospitalization expenses.

According to Galan et al. [16], pulmonary contusion could be found in about 75 % of flail chest patients. Pulmonary contusion, which leads to pulmonary vasoconstriction and thereby shunt and mismatch, is one of the main factors that could induce respiratory distress in these patients. Voggenreiter et al. [17] found that surgical treatment for flail chest patients with pulmonary contusion did not significantly reduce ventilation time and ICU stay, which could be caused by the presumption that hypoxemia and respiratory distress are mainly caused by pulmonary parenchymal injuries induced by pulmonary contusion, not by paradoxical breathing. The findings of the present study showed that for flail chest patients with pulmonary contusion, shorter ventilation time was needed in patients who underwent surgery compared with those who received conservative treatment. We propose that paradoxical breathing could not only induce mediastinal swing and influence the circulation system but also greatly decrease tidal volume [2], which could be improved by surgery.

Pulmonary infection is a common complication during flail chest treatment. Studies have reported that pulmonary infection is one of the main factors associated with longer time of mechanical ventilation and ICU stay, as well as with poor prognosis [18]. In the present study, the rate of pulmonary infection was significantly lower in the surgical group compared with the conservative group. This could be explained, at least in part, by the following reasons: 1) early ventilator weaning could effectively decrease the incidence of ventilator-associated pneumonia; 2) early ventilator weaning allows early ambulation, physical exercise therapy, and autonomous cough and expectoration, which could reduce the accumulation of airway secretions, and prevent hypostatic pneumonia and even lobar atelectasis. As previously shown, the requirement for tracheostomy and endotracheal re-intubation could increase in patients needing long-term mechanical ventilation or for patients with weaning difficulties [19, 20]. Therefore, since surgical treatment of flail chest is associated with a shorter requirement for mechanical ventilation, surgery should decrease the need for tracheostomy and endotracheal re-intubation.

APACHE II score is a reliable parameter for the evaluation of condition severity in critically ill patients [14]. In the present study, no significant difference in APACHE II score was found between the two groups at admission and on the seventh day after admission. However, the scores were statistically different (in favor of the surgical treatment group) on the 14th day after admission between the two groups. As the mean time between trauma and surgery was 6.5 days in the present study, these findings could further confirm that surgical treatment could lead to better outcomes compared with the conservative treatment. The improvement of the overall condition could also directly reduce the treatment cost. Bhatnagar et al. [21] also reported that although additional costs were needed for surgical treatments, the overall hospitalization expenses could still be lower than the expenses for the patients in the conservative treatment group.

The time of ICU stay was significantly shorter in the surgical group compared with the conservative group, which was in accordance with our results about shorter ventilation time, lower incidence of pulmonary infection, and better overall condition improvement in the surgical group compared with the conservative group. A meta-analysis in flail chest patients [10] also demonstrated that surgical treatment could shorten the ICU stay by about 3.4 days compared with a conservative treatment.

The study by Voggenreiter et al. [17] showed that for patients treated with surgery within 48 h after trauma, the average time to tracheal extubation was 6.5 days. In the present study, results may suggest that an early operation could result in a shorter mechanical time (7.9 days), ICU stay (12.1 days), and therapeutic time of antibiotics (10.4 days) compared with patient who underwent a late surgery (12.3, 18.6, and 18.3 days, respectively). As is shown on Fig. 1, one patient with an early surgical fixation was extubated on postoperative day 3. In addition to being a retrospective analysis, the present study may suffer from additional limitations. First, the sample size was relative small. Finally, the understandings of the indications for surgical treatment were different among different clinicians. Therefore, further large multicenter studies are required to answer this issue.

**Fig. 1:** **a**–**b** Fifty-five-year-old patient (the surgery group) sustaining anterolateral flail chest due to segmental fracture of ribs 4–9, hematopneumothorax, pancreatitis, rupture of the spleen. **c** Endotracheal intubation and insertion of a chest tube immediately after entering ICU. **d** Chest wall stabilization of ribs 3–6 was performed 4 days after admission and extubation at the third day after surgery

## Conclusions

In summary, internal fixation could be a good treatment approach for severe flail chest, providing early stabilization of the loose thoracic wall, correction of paradoxical breathing, reduction of the time of mechanical ventilation and ICU stay, decreasing the possibility of pulmonary infection, and prevention of residual thoracic deformities and subsequent long-term effects on pulmonary function.
